# Sports Economic Mining Algorithm Based on Association Analysis and Big Data Model

**DOI:** 10.1155/2022/1518202

**Published:** 2022-05-23

**Authors:** Fujian Zhou

**Affiliations:** School of Law, Guangdong Peizheng College, Guangzhou 510800, China

## Abstract

With the implementation of national strategies such as sports power and national fitness, the sports economy has become an important element of high-quality national development, and the demand for sports economy and management talents is greatly increased. Particularly in the new area with big data as the typical feature, the teaching content, teaching method, and teaching mode of sports economics and management majors have put forward new requirements. The continuous progress of storage and network technology has prompted the generation of massive multisource spatiotemporal data in various fields. The advantage of association analysis algorithms is that they are easy to code and implement. The relationships found by association analysis can take two forms: frequent itemsets or association rules. We use correlation analysis methods to perform correlation learning between sports economy and related big data and thus improve the development of sports economy. Mining and analyzing the relevant big data can precisely reveal the problems of sports economic development and can realize the fine management of sports, thus contributing to the healthy development of sports. Mastering the skills of acquiring, analyzing, and applying big data is the core content of sports economic analysis. The sports economy has refined and intelligent management means, and its adoption of virtual reality reflects the current situation and development trend of the sports business, which further highlights the status and role of multisource big data in the sports economy. Based on these, this paper proposed a sports economy mining algorithm in view of the correlation analysis and big data model. Then, we verified the effectiveness of the model through experiments, which laid the foundation for the development of the sports economy.

## 1. Introduction

The major of sports economics and management is a cross-cutting emerging discipline that studies sports economic issues. The major cultivates professionals who are familiar with the basic theories of kinesiology and economics, master the basic methods of economic analysis, and engage in economic analysis of the sports market, sports career planning sports economic management, and sports science research [1]. As sports economic issues become a hot issue in social development, the major of sports economics and management has also achieved rapid development, but there are still many shortcomings in the curriculum and practical teaching, and the future should focus on internal construction and innovative teaching mode. Practical application is an outstanding feature of the major [2]. With the change of network technology and economy and world, the actual needs of society have changed, among which the sports industry business has changed greatly, the network (online) economy accounts for more and more, and network technology and big data mining analysis should become an important content and means of sports economics and management [3]. However, at present, there is not much involvement in network technology, especially big data mining analysis. The teaching of sports economics and management causes a serious disconnect between the cultivation of talents' skills and social needs.

In the area of big data, sports economics and administer talents are required to be able to find the key in the huge amount of sports big data and to be able to use big data analysis software and methods to solve problems encountered in sports economic development, sports event management affairs, and stadium operation [4]. This requires that the teaching of sports economics and management should have broader professional knowledge and a more optimized curriculum structure. The analysis of the sports big data needs to be practiced continuously in practice, while most of the current teaching of sports economics and management majors does not provide a practice platform that meets the actual needs, not to mention the understanding and processing of complex problems, which makes the talents cultivated by colleges and universities unable to meet the needs of world change. Therefore, it is essential to fully recognize the various problems of teaching sports economics and management majors and give precise solutions. The following big data knowledge should be included in the education of sports economics and administered in the new era: first, to master the theoretical knowledge of relevant networks and big data; second, to understand the types and structures of big data of sports economy; third, to master the collection and processing methods and software of big data of sports economy; fourth, to be able to solve real-life problems through analysis [5].

The era of big data will bring revolutionary changes to data collection and utilization, analysis methods, and research tools in the field of teaching and research of physical education disciplines. Multisource big data is an important basis for objectively understanding sports systems and summarizing their development laws. Big data is based on refined individual activity data. In order to grasp the operation and management rules of sports, big data can analyze and predict different sports fields, establish big data models, conduct quantitative simulations, and guide decision-making on practical problems. The main contributions of this paper are as follows: (1) Research on the acquisition and analysis techniques of sports big data is beneficial to the theoretical study of sports economics and management teaching, enriching the discipline system, expanding the discipline direction, and enhancing the applicability of the knowledge structure of cultivated talents. (2) Research on the analysis methods and techniques of big data is an effective way to improve the teaching quality and practicality of sports economics and management. (3) This paper proposes a correlation analysis and big data model of sports economy mining algorithm and verifies the effectiveness of the model through experiments, which lays the foundation for the development of sports economy.

## 2. Related Work

### 2.1. Current State of Research on Association Analysis

In general, association analysis, or association mining, usually refers to the traversal of transactional data, relational data, or other data carriers to mine frequent patterns or causal structures between items, between sets of items, or between sets of items. Association analysis algorithms can usually be divided into three main categories from the perspective of the data structures processed. Association algorithms are based on a priori knowledge and horizontal data format. This class of algorithms is represented by the Apriori algorithm, which usually uses a layer-by-layer iterative search to mine the relationship between sets of items in the database to form rules, and its process specifically includes joining and pruning. Represented by Eclat and CHARM, unlike the previous two algorithms, this class of algorithms uses a vertical data format and is based on depth-first, refining the search space into smaller subspaces using prefix-based hierarchical relations based on conceptual lattice theory [6]. Represented by FP-growth, this class of algorithms usually maps the database in a specific form (e.g., FP-tree, with the structure illustrated in Figure 1) to avoid repeatedly traversing the original database.

However, the above three classical association analysis algorithms have the following problems: all three association analysis algorithms are based on a common minimum support framework; that is, the application decision-maker needs to artificially set minimum support to ensure that frequent itemsets can be filtered out in each iteration, which follows the a priori property, also known as the downward closure property, that any subset of frequent itemsets must be frequent [7]. The above minimum support framework also poses an important problem for the application of the algorithm: in order to be able to propose suitable minimum support, the decision-maker needs to have sufficient goal knowledge and detailed prior knowledge about the target task and to be able to accurately predict the number of rules to be generated before the mining work is completed [8]. In addition, the minimum support setting itself is very delicate; if it is set too small, the algorithm will return a large number of frequent patterns, most of which may be a priori stale knowledge or uninteresting mining results; if it is set too large, the algorithm may fail to generate patterns [9].

In addition, the frequent itemsets returned by classical correlation analysis algorithms tend to contain a large amount of common empirical knowledge; that is, they do not provide new, valuable knowledge [10]. At the same time, the minimal support-based framework determines that it is likely to miss frequent patterns that occur less frequently but are extremely valuable. To solve this problem, efficient mining becomes an effective mining tool, which discards the traditional minimum support framework by setting the utility of each item and pruning the filter using the minimum utility value. Here, utility refers to the degree of importance of a particular item [11].

### 2.2. Current Research Status of Big Data Knowledge Self-Organization Model

As far as the current situation of domestic research is concerned, the research on knowledge self-organization mainly focuses on the research on information self-organization and the research on data self-organization, highlighting three aspects: the causes of knowledge self-organization, the application of knowledge self-organization, and the law of motion of knowledge in knowledge self-organization [12]. In today's society with the rapid development of the Internet, the transmission of information is not limited to paper, telephone, and other methods, and the network information transmission methods are diversified. Network information self-organization is in a specific functional area, the network without external instructions to organize information on their own, automatically from disorder to orderly process, network information self-organization has a variety of manifestations, and the use of the construction of the platform is a key factor to effectively realize the self-organization of information [13]. Relevant researchers have mainly studied and discussed the phenomenon of knowledge self-organization in science and technology information systems, giving a definition that refers to a process in which, under certain conditions, the elements within knowledge interact with each other and move according to certain laws to form a new structure. They analyze the self-organization conditions that satisfy the system, so that the entire S&T information system is constantly coordinated and selected through the role of feedback, forming new characteristics to adapt to the changing environment while adding value to S&T information in coordination and increasing its effectiveness [14]. The structure diagram of the big data knowledge self-organization model is shown in Figure 2.

Figure 2 contains five main modules, which are event and corresponding rule input, intelligent comparison, chunking, and result output. The most important of them is the intelligent comparison. In the study of knowledge self-organization, most of the scholars have recognized the knowledge self-organization characteristics of knowledge in the network environment and have exploratively proposed the basic theory and methods of network knowledge self-organization in development, management, and operation. In the process of studying the research mechanism of knowledge self-organization in the network, it is difficult to form a system, and thus no systematic analysis or proof can be made [15]. There are two main reasons for this situation. First, network information and network knowledge and modern self-organization theory were generated almost in the same period, both are in the stage of rapid development, and neither of them has established a relatively perfect knowledge system and theory system. Second, the generation, dissemination, and utilization of network information and knowledge must be supported by new technologies on the network [16]. However, the knowledge self-organization system is in a complex network system, and there are many factors affecting its development, such as environment, humanities, and many other factors. Therefore, if we want to apply the self-organization theory in natural science in the process of knowledge organization, we will encounter more environmental and systemic factors.

### 2.3. Current State of Research on Data Mining Models

The core of big data analytics is data mining algorithms. From a professional view, data mining is the use of a series of relevant algorithms and techniques to extract the information and knowledge needed from a large amount of data. It can help decision-makers extract potential relationships and patterns in the data through the analysis of historical and current data and help them predict possible future situations and upcoming results [17]. Data mining algorithms have been relatively mature in dealing with data of modest size. Some classical algorithms, such as clustering algorithms, classification algorithms, and association rule algorithms, have been widely used in practice [18]. However, with the growth of the data process, previous mining algorithms are no longer suitable for handling big data, although there has been research on mining algorithms for massive data, such as mining algorithms based on random sampling, mining algorithms based on distribution, and mining algorithms based on incremental [19]. These algorithms improve the traditional mining algorithms to some extent and make them capable of handling massive amounts of data, but the results are still not ideal in the face of ever-growing data.

At present, there is not much research on data mining algorithms for big data at home and abroad, but the mining algorithms for handling smaller data volumes are well established. Data mining has been researched and developed for decades, resulting in a wide variety of data mining algorithms. The emergence of distributed computing provides a new direction for processing and analyzing massive amounts of data. Distributed computing means that many software share information [20]. This software can run either on the same computer or on multiple computers connected through a network. Distributed calculating processes the data distributed on each node and merges the processing results according to certain rules, which can solve the memory limitation question and improve the mining efficiency at the same time. Nowadays, cloud computing has emerged to provide a new platform for distributed mining [21]. Cloud calculating can distribute computing tasks across many interconnected machines, enabling various applications to access computing resources, storage resources, and other service resources on demand. For cloud computing, people's research is mostly focused on the parallelization improvement of traditional data mining algorithms so that they can be computed on cloud platforms, there has not been a major breakthrough yet, and deeper research is still needed [22].

Incremental data mining is to divide data into different data blocks through certain data segmentation methods and then perform data mining on each data block in turn, where the mining of the current data block depends on the mining results of the previous data block. Similarly, the incremental mining method effectively solves the problem of memory limitation due to the approach of dividing the data [23]. Due to the large amount of data processed each time, the running time is reduced, and the efficiency is improved [24]. Therefore, the research based on incremental mining algorithms has also become one of the important directions for processing and analyzing huge amounts of data. From the incremental data mining process, it is easy to see that how to more effectively use the already mined results to mine the later data is one of the factors that affect the effect of the final mining.

## 3. Basic Principles and Concepts of Algorithm

This section provides an introduction to the data association analysis model and the big data model, mainly focusing on the concepts and fundamentals of the two algorithms after the conclusion of the case.

### 3.1. Basic Principle of the Correlation Analysis Algorithm

Nowadays, one of the topics in big data research is data mining. Therefore, continuous attribute discretization is also one of the main focuses of scholars' research at this stage. There are many different types of discretization algorithms, each with its own characteristics, but the core of the discretization algorithm is the same; that is, the selection of the best cutting and merging points is the key in the process of discretization operation, which is also the difficulty and focus of the research of discretization technology at this stage [20]. When preprocessing data, the most suitable discretization method should be selected according to the characteristics of data existence.

Before introducing the discretization algorithm, let us first introduce the knowledge that is frequently used in the discretization algorithm. Entropy is a concept in physics that is usually used to describe the degree of the chaos of a molecule. Drawing on the idea of thermodynamic entropy, the concept of information entropy is proposed to measure the average uncertainty in information systems. The formula for calculating information entropy is shown as follows:

(1) $$\begin{array}{c} H\left(X\right)=-\sum_{x}p\left(x\right)\log\;p\left(x\right)=-\sum_{i=1}^{n}p\left(x_{i}\right)\log\;p\left(x_{i}\right). \end{array}$$

In equation (1), *x* is a randomly selected discrete variable and *p*(*x*) is the probability of occurrence of *x*. The choice of the log function base is arbitrary and is the information entropy of the random variable *x*. A larger value of information entropy indicates a higher degree of confusion in this dataset. Then comes the conditional entropy. In simple terms, the conditional entropy represents the information entropy of *Y*, or the uncertainty of *Y*, given a particular condition *X*. Its formula can be expressed as follows:

(2) $$\begin{array}{c} H\left(Y|X\right)=\sum_{x}p\left(x\right)H\left(Y|X=x\right)=-\sum_{x}p\left(x\right)\sum_{y}\left(yx\right)\log\;p\left(yx\right). \end{array}$$

Conditional entropy can also be defined as the mathematical expectation of the conditional probability distribution of *Y* with respect to the precondition *X* under a particular precondition *X*. One point of interest when calculating the information entropy gain is that the information entropy to be classified is unknown [21], so the computational formula usually uses the empirical entropy or empirical conditional entropy calculated from the sample. There are numerous discretization algorithms for continuous features of the general process handled by the discretization method, but they generally go through the following steps for processing. The general steps of correlation analysis are shown in Figure 3.

The first is sorting. In the case of a huge amount of data, sorting the data before running the discretization algorithm improves the efficiency of the discretization algorithm, reduces the time needed to run the discretization algorithm, and decreases the time complexity and space complexity compared to the disorderly order [22]. Then comes the selection of a cut point. A point in the data interval is selected as the cut point, and the criterion for measuring the cut point developed in the discretization algorithm is used to judge whether the point satisfies the cut criterion in the discretization algorithm. If the selected cut point satisfies the measure in the discretization algorithm, the dataset is sliced or merged, and the next step is performed. When there is a stop condition in the discretization algorithm, the discretization process is stopped when the stop condition is satisfied, and if not, it is run until the condition is satisfied, resulting in the final discretization result. The same dataset using different discretization algorithms will produce different discretization results. When performing discretization operations, the ideal state is to maximize the retention of the attribute intervals represented by the decision information while being as parsimonious as possible. The basic principle of discretization is to compress the data by using the hidden laws in the data, which belongs to the inductive reasoning method, and it can be said that when the amount of data is larger, the amount of information obtained from the data will be larger [23].

### 3.2. Basic Principle of Big Data Algorithm

Incremental clustering is mostly used for streaming data. For dynamically increasing data, it is obviously too expensive to recluster these data together with existing data, especially for large datasets. Moreover, the information on existing data clustering is not effectively used, resulting in a great waste of computational resources [25]. A reasonable and effective way is to use the clustering results of the existing data to cluster the new data, which is the basic idea of incremental clustering. Point-by-point incremental clustering means that each new data is added with only one data point, which is obviously not applicable to large data because it causes frequent clustering and makes clustering inefficient. Block-by-block incremental clustering means that each new data is a collection of data points, which ensures that the amount of data processed does not exceed the memory limit and does not call too many clustering algorithms [26].

FCM is one of the useful fuzzy algorithms, which is a process of clustering by assigning different weights to the data points according to their importance. The algorithm first randomly selects *k* different initial clustering centers and calculates the affiliation of each data point according to equation (3). Then, it updates the clustering center according to equation (4), recalculates the affiliation of each data point after getting the new clustering center, and repeats the process until the result is reached.

(3) $$\begin{array}{c} u_{j}=\sum_{l=1}^{k}{\left(\frac{d_{ji}^{2}}{d_{l}^{2}}\right)}^{\left(-1/m-1\right)}. \end{array}$$

In equation (3), *d*_*ji*_^2^ denotes the distance between *i* and *j*, *d*_*l*_^2^ denotes the size of *l*, and *m* is the number of confusions.

(4) $$\begin{array}{c} v_{j}=\frac{\sum_{i=1}^{n}\omega_{t}u_{j}^{m}x_{i}}{\sum_{i=1}^{n}\omega_{ı}u_{\mu }^{m}}. \end{array}$$

When clustering a linearly indistinguishable dataset, the clustering result of WFCM is less accurate, and then the data points can be mapped to a space by the method of kernel function to make the data linearly distinguishable. The WKFCM algorithm is a clustering method based on the WFCM algorithm, which maps data to a high-dimensional space by means of a kernel function. The kernel function is defined in equation (5).

(5) $$\begin{array}{c} k\left(x_{t},x_{j}\right)=\Phi {\left(x_{t}\right)}^{T}\Phi \left(x_{j}\right). \end{array}$$

WKFCM and WFCM processes are basically the same; the difference is the distance calculation formula. In WKFCM, the distance is defined in equation (6).

(6) $$\begin{array}{c} d_{ji}^{2}=\Phi \left(x_{i}\right)-\Phi {\left(v_{j}\right)}^{2}=k_{ii}+k_{ji}-2k_{ji}. \end{array}$$

And the update formula of the clustering center is shown in equation (7).

(7) $$\begin{array}{c} \Phi \left(v_{J}\right)=\frac{\sum_{i=1}^{n}\omega_{1}u_{jl}^{m}\Phi \left(x_{i}\right)}{\sum_{i=1}^{n}\omega_{t}u_{ji}^{m}}.\; \end{array}$$

It should be noted that since there is no specific expression in the mapping function, it is not possible to find the specific value of the clustering center vector in the WKFCM algorithm. A central step in the simplicity of the incremental clustering model is the exploitation of the clustering results of existing data blocks, and a number of improved algorithms have been developed to address this problem. The incremental kernel fuzzy clustering algorithm is the process of continuously reclustering the new data blocks and the result of own clustering, and its clustering is the same at each step. Incremental clustering is an extension of the ordinary clustering algorithm, and some defects of the ordinary clustering algorithm still exist in incremental clustering, such as the number of clusters that needs to be specified in advance and sensitivity to the initial cluster centers, which have an impact on the clustering accuracy. This method of selecting the initial clustering centers takes into account the data characteristics of the additional data while maximizing the use of incremental clustering. The principle is shown in equations (8) and (9).

(8) $$\begin{array}{c} V_{t-1}=\left\{v_{1}^{t-1},v_{2}^{t-1},\ldots ,v_{k}^{t-1}\right\}\\ d_{ij}^{v}=\Phi \left(v_{t}^{t-1}\right)-\Phi \left(v_{j}^{l-1}\right). \end{array}$$

The clustering center update formula is shown in equation (9).

(9) $$\begin{array}{c} v_{j}^{t-1}\leftarrow \frac{\omega_{j}f_{j}\left(V_{t-1},x_{t}^{t}\right)+x_{i}^{t}}{\omega_{j}+1}. \end{array}$$

Its corresponding weight update formula is shown in equation (11).

(10) $$\begin{array}{c} \omega_{J}\leftarrow \omega_{j}+1. \end{array}$$

In the second stage, new data structures are discovered by processing the data points in the process. A simple distance-based method is applied in this stage. The conceptual diagram of the model is shown in Figure 4.

Using the clustering results of the already clustered data is the core of incremental clustering. Incremental clustering requires the transfer of clustering information to subsequent data blocks, and the data points that carry this information are called transfer points. In many incremental clustering algorithms, the transfer points are generally selected as cluster centroids, and only one transfer point is selected for each class of information; that is, this one transfer point is considered to contain all the information of the class. However, when data points belonging to different classes are incorrectly classified into one class, and then the transfer point will pass the wrong clustering information to the subsequent data blocks, affecting the final clustering accuracy. And this wrong information is difficult to be corrected in the subsequent clustering process. In addition, when the amount of data is relatively large, one transfer point does not contain all the information of the class, which makes the clustering information lost in the transfer process.

## 4. Sports Economic Mining Algorithm

This session provides a detailed description of the data mining algorithm for sports and athletics, focusing on two aspects of data traceability and big data fusion model.

### 4.1. Data Traceability

Data traceability is a relatively new research area, and there is no uniform definition in the computer field. Initially, some literature called it data archives or data logs, and later most of the literature called it data origins, which is used to trace the origin and generation process of data. The core of data traceability is traceability metadata, and any traceability system needs to manage its traceability information well, which necessarily requires an overall traceability framework. In this section, a tag-based fine-grained data traceability method is proposed, which is mainly an extension of traditional Hadoop, and it mainly includes automatic capture mechanism of traceability information, traceability tag storage, and traceability tracking method.

This section will first analyze the internal execution principle of MapReduce, propose its own design ideas, and finally implement its traceability capture. A MapReduce task is broadly divided into two tasks, a Map Task and a Reduce Task, and each task corresponds to several different phases. The Map Task process mainly includes the *recordreader* stage, mapper stage, and the *ipartition* process for mapper output, as shown in Figure 5.

Through the above analysis of *MapReduce* processing flow, this paper will extend the *MapReduce* framework on top of it and use a wrapper-based approach to dynamically add and capture traceability tags during workflow execution without affecting its parallel execution and fault tolerance. *MapReduce* is the most commonly used technology for data processing under big data platforms, and in the actual model workflow, the processing nodes can include big data processing technologies such as spark real-time computing framework.

### 4.2. Big Data Fusion Model

In view of the problem that the data is huge and noisy and not easy to manage in the massive data environment, this paper fully analyzes the data characteristics of big data and proposes the research of big data fusion model method based on tensor half-tensor product. Currently, there are corresponding representation models in some specific domains, but they can only be applied to a specific domain and cannot be generalized to all big data, and the representation methods of these models are not complex enough to represent massive high-dimensional data uniformly. After encoding the massive high-dimensional data, the data is divided into the original data part and the scalable part, and the uniform tensor representation model is defined as follows:

(11) $$\begin{array}{c} T\in R^{I_{t}\times I_{s}\times I_{c\times }I_{1}\times I_{2}\times \ldots \times I_{p}}. \end{array}$$

In this tensor model, each different order of the tensor represents a different attribute of the data. For example, the attributes such as width and height as well as color and time of the video data are extracted and then converted into different orders of the tensor and then added to the base tensor space. To achieve the tensor expansion, the tensor expansion operator based on the half-tensor product is defined as follows:

(12) $$\begin{array}{c} X\propto Y_{:}=\sum_{i=1}^{m}X^{i}y_{i}\in R^{n}. \end{array}$$

In the real situation, the structured, semistructured, and unstructured multisource heterogeneous data are first represented as subtensor models of lower order, and then the heterogeneous data can be first represented as low-order subtensor using tensor expansion operators so as to achieve a unified representation of various data. When the orders of two tensors have the same properties, they can be combined by tensor expansion, and those orders with different properties are to be preserved. The basic structure block diagram of the data fusion algorithm is shown in Figure 6.

## 5. Experiments and Results

We conducted the experiments in the following hardware and software environments, specifically (1) Windows 10 system platform. The relevant configurations of the experimental platform are as follows: (2) processor is Intel(R) Corei5; (3) RAM memory is 32.0 GB; (4) system type is 64-bit OS. We use a data sample containing 100 samples, of which 80 are training sets and 20 are test sets. The detailed training method is as follows: the batch size is set to 8, the batch size is the size of the selected training sample and the limitation of the device GPU, and the best optimization and speed are selected according to the model. The initial vector of the model is set to 0.0001; the Adam optimizer is used. The time-series data caliber selected in this paper is 1994–2015, and two indicators, TYTR (financial investment in sports) and GDP (gross regional product), are used for analysis. Among them, the data of financial investment in sports from 1994 to 2003 were obtained from the Journal of Zhangjiakou Finance; the data of financial investment in sports from 2004 to 2015 were obtained from the annual financial account reports of Zhangjiakou Finance Bureau; the data of GDP of Zhangjiakou from 1994 to 2003 were obtained from the Study on the Analysis of Regional Economic Differences and Coordinated Development in Hebei Province. At present, financial investment is the main source of funding to support the development of local sports in Zhangjiakou. As the government of Zhangjiakou attaches more and more importance to the development of sports, the financial department has also continued to strengthen financial support for the development of sports industry, which has also greatly promoted the development of local sports.

To perform the long-run equilibrium relationship test, the prerequisite is that the time-series data must be guaranteed to be stationary. In this paper, the ADF unit root test is firstly used to test the smoothness of LNGDP and LNTYTR, and the test results are shown in Table 1. The initial data of DLNTYTR and DLNGDP cannot reject the original hypothesis of the existence of unit root at the 5% test level; that is, the initial data of LNTYTR and LNGDP are not smooth.

From the above test results, it can be seen that Zhangjiakou's sports financial input and regional GDP have passed the smoothness test, so cointegration test can be conducted. This paper uses the Engle-Granger two-step test to test the long-run equilibrium relationship between the amount of financial input to sports and the regional GDP of Zhangjiakou. Finally, the same method ADF unit root test is applied to test the stationarity of ECM, and only when the residual ECM belongs to the stationarity series, can it show that the long-run equilibrium relationship between the financial input of sports and the regional GDP of Zhangjiakou is established. As can be obtained from Table 2, the residual ECM rejects the original hypothesis of the existence of unit root at the 5% test level; that is, the residual series is smooth, which means that the long-run cointegration relationship between the financial investment in sports and the regional GDP obtained earlier can be established. Moreover, in the long run, every 1% increase in financial investment in sports can lead to a 0.6074% increase in regional GDP.

In the process of constructing the VAR model, the key is the selection of lags. Generally, the lags of variables are determined according to the principles of AIC and SC minimization, but when the lags corresponding to the minimum values of AIC and SC are different, the selection can be made according to other principles such as the deficit pool, information criterion, and LR and HQ statistics.  Table 3 shows the construction of the VAR model of financial investment in sports and regional GDP in Zhangjiakou. The lags should be determined in the same way as in the VAR model, so the lag of the ECM should also be 1. From the results of the error correction model estimation, it can be concluded that the goodness of fit of the model is 57.52%, and the T and F statistics pass the significance test.

This indicates that the increase of financial investment in sports does not lead to the increase of local GDP. In conclusion, the increase of regional GDP can promote the increase of financial investment in sports, but in turn, the increase of financial investment in sports will not promote the increase of regional GDP. The degree of shock contribution between financial investment in sports and regional GDP in Zhangjiakou is shown in Figure 7.

As can be seen from Figure 7, the horizontal coordinate indicates the number of training rounds, the vertical coordinate indicates the performance, Zhangjiakou's regional GDP is only affected by its own fluctuation shock in period 1, but not by financial investment in sports, and the degrees of contribution of its own shock and financial investment in sports are 100% and 0%, respectively; it keeps decreasing in periods 2–10 by its own shock, but the decrease is small. The impact effect of financial investment in sports on regional GDP started to appear from the 2nd period and began to rise, but the rate of increase was slow. From the 1st period, the financial input of sports is affected not only by its own fluctuation but also by the impact of regional GDP, but the impact effect of regional GDP is not yet obvious; at this time, the contribution of financial input of sports to the impact of itself and regional GDP is 99% and 1%, respectively. In the 2nd–10th period, the degree of contribution of GDP to the impact of financial input of sports business increases at a faster rate, the impact effect by itself decreases continuously, and the degree of contribution of both to the impact in the 10th period is 36% and 64%, respectively, which indicates that the financial input of sports business in Zhangjiakou is stronger by the impact effect of GDP.

## 6. Conclusion

The added value of China's sports industry output has been rising year by year and has formed a complete industry chain of upstream resource production, midstream industry operation and dissemination, and downstream product arrival while integrating new industries to form new economic benefit growth poles, but there is a big difference with the economic development of sports industry in developed countries. In particular, it is very obvious. Secondly, the structure of China's sports industry is at the low end of the industry and a low degree of marketization. This paper proposes a sports economy mining algorithm based on the correlation analysis and big data model and verifies the effectiveness of the model through experiments, which lays the foundation for the development of the sports economy.

The new field, typified by big data, has put forward new requirements for the teaching content, teaching methods, and teaching modes of sports economics and management majors. The continuous progress of storage and network technology has prompted the generation of a large amount of multisource spatiotemporal data in various fields. The advantage of association analysis algorithms is their ease of coding and implementation. The relationships discovered through association analysis can take two forms: frequent itemsets or association rules. The mining and analysis of relevant big data can accurately reveal the problems of sports economic development, which can realize the fine management of sports and thus promote the healthy development of sports. With the development of China's sports industry, the growing number of people who participate in exercise has led to a steady increase in the size of the sports consumption market. Physical sports consumption in the traditional sense has been breaking through with the boundary of the sports industry's industry update and Internet technology, and more sports services, experiences, and even virtual products have started to be included in the scope of sports consumption. Big data of tournaments enables information sharing through online platforms and obtains information feedback through people's comments and retweets. Globally, using big data to analyze the type and distribution of sports events, organization, and management, evaluation and effects of sports events and changes in the scale of sports events and the trajectory of individual participants will be an inevitable trend in the future. In the future, we plan to start using recurrent neural networks for correlation analysis and identification [27].

## Figures and Tables

**Figure 1:** FP-tree structure diagram.

**Figure 2:** The structure diagram of the big data knowledge self-organization model.

**Figure 3:** The general steps of correlation analysis.

**Figure 4:** The conceptual diagram of the model.

**Figure 5:** Block diagram of the structure of Map Task.

**Figure 6:** Block diagram of the basic structure of the data fusion algorithm.

**Figure 7:** The contribution between financial investment in sports and GDP.

**Table 1:** Stability test results.

Variables	Inspection form	ADF statistics	Critical value	Conclusion
LNGDP	(C, T, 1)	−0.40	−3.020	Unstable
DLNGDP	(C, T, 0)	−3.18	−3.029	Stable
LNTYTR	(C, T, 0)	0.76	−3.012	Unstable
DLNTYTR	(C, T, 0)	−4.43	−3.020	Stable

**Table 2:** Residual smoothness test results.

Variables	Inspection form	ADF statistics	Critical value	Conclusion
ECM	(C, T, 1)	−3.40	−3.050	Stable

**Table 3:** Construction of the VAR model.

Lag period	LogL	LR	FPE	AIC
0	−27.88568	87.10384	0.094904	3.320631
1	24.37663	1.479517	0.000448	−2.041847
2	25.40091	3.232753	0.000638	−1.711212
3	28.04589	6.020715	0.000785	−1.560654

## Data Availability

The datasets used during the current study are available from the corresponding author upon reasonable request.
